The article "Study on the Practice of Enterprise Financial Management System under the Epidemic Norm Based on Artificial Neural Network" was retracted in 2024. Reasons: signs of a paper mill; suspected computer-generated content; unreliable results or conclusions; concerns about the data.

# Study on the Practice of Enterprise Financial Management System under the Epidemic Norm Based on Artificial Neural Network

**DOI:** 10.1155/2022/7728596

**Published:** 2022-09-06

**Authors:** Kaiheng Ji

**Affiliations:** Edinburgh Business School, Heriot-Watt University, UK

## Abstract

The sudden arrival of the new crown epidemic has had a significant and long-lasting impact on the division's economic environment as well as the production and operation activities of businesses. As far as the financial management is concerned, opportunities and difficulties are faced by enterprises of all types. With reference to the available research data, enterprises have an important contribution to GDP and jobs, but they still face a series of difficulties and challenges in their development in the context of the normalization of the epidemic. By analyzing the impact of the new crown pneumonia epidemic on the financial management work of enterprises, this paper proposes an artificial neural network-based enterprise financial forecasting and early warning method to provide an effective method for enterprise financial management. For the time-series characteristics of enterprise finances, a prediction model based on long- and short-term memory networks is developed which acknowledges the necessity of combining the temporal dimension with the spatial dimension for forecasting. This model incorporates time qualities into the data to the existing forecasting model. It also considers both working and nonworking day data and thoroughly considers the factors influencing corporate finance. Then, using BP neural network for financial risk prediction, nonfinancial index factors should be added to the financial early warning model thus eliminating the limitations of the financial early warning model. At the same time, the accuracy of the prediction can be improved which is more suitable for enterprises to apply in practice. The experimental results demonstrate that the financial prediction model built by multilayer feed forward neural networks and recurrent neural networks based on error back propagation training is inferior to the prediction model built by long- and short-term memory network. Regardless of the degree of fitting or prediction accuracy, the BP neural network model outperforms the conventional model for enterprise financial warning. Under the normalization of the pandemic, the combined use of both can offer an efficient technique for enterprise management.

## 1. Introduction

Globally, the level of epidemic is accelerating the deconstruction of the original world pattern. The global economy is in deep recession, and economic globalization is encountering counter current. The protectionism and unilateralism are in full swing forcing enterprises to seek survival and development in an environment of higher uncertainty.

The new epidemic of 2020 will result in the slowing down of economic growth. In addition to this, the tensions in trade between China and the U.S. contribute those factors which brings difficulties and opportunities for Chinese business and enterprise. On the one hand, enterprises are trying to survive dealing with unfavorable circumstances including decreased demand, declining revenue, and limited cash flow, as well as the serious issue of a disruption in the global supply chain and industrial chain. On the other hand, China has been pushed to speed up industrial upgrading due to the outstanding outcomes of epidemic prevention and control and the economic recovery brought about by trade fictions [1]. It further enhances the major strategic deployment at the national level and improves digital technology to bring new dynamic energy and provides a series of important opportunities. It helps enterprises to find opportunities in the crisis and seek development in difficulties [2]. Financial management is related to the lifeline of the whole enterprise, especially in the complex and changing economic environment, challenges, and opportunities. It is urgent to innovate and upgrade the enterprise financial management model and build a response strategy for enterprise financial management in the postepidemic era.

As a major public health emergency, the Newcastle pneumonia epidemic will undoubtedly bring significant impacts and challenges to economic development [3]. The impact of the epidemic on economic activities is mainly reflected in the following five aspects as shown in Figure 1.

- Consumer demand shock: the new crown pneumonia epidemic has brought a serious impact on the consumer demand of residents [4]. Unemployment, shopping inconvenience, and wait-and-see mood will cause the consumer demand of residents to drop in the epidemic area
- Labor supply shock: similarly, a high unemployment rate brought on by an epidemic also aids in its further spread. This results in the increase of economic and social pressure on those who are unemployed
- Shocks to the supply and demand structure: during the epidemic, the number of illnesses and deaths increases rapidly. People resort to home quarantine to avoid the risk of infection. This results in a sharp decline in labor supply. As a result, some sectors of the economy that are severely affected by the epidemic cease operations. This leads to a more severe crisis in labor supply and consumer demand [5].
- Impact on regional GDP: sudden epidemics affect the stability of the economic system and impede the growth of regional GDP
- Shocks to the world's commerce and economic systems: the first wave of the epidemic will cause closures and disruptions in national supply chain in areas that serve as the hubs of these networks. This creates production and consumption crises. The second wave will spread infections in more countries which will have the short-term effects of stifling economic expansion, escalating market fear, and raising financial dangers

Traditional enterprise management places more emphasis on the analysis of enterprise development strategy while ignoring the analysis of enterprise financial management and risk mitigation. This makes it difficult for enterprises to respond quickly when they encounter serious issues [6]. According to numerous real-world examples, financial crises frequently precede enterprise crises. Financial forecasting and early warning models are used to identify hazards and notify managers of various issues so they can find them and address them quickly. These models are built using a variety of information including financial reports, audit reports, and company disclosures.

The high growth and high risk characteristics of enterprises determine that the energy market has a large risk in operation process [7]. Many financial risks do not break out suddenly and can be reflected by financial data in the early stage. The research on financial management of enterprises under the epidemic norm is not ideal even though there are more studies on financial early warning. According to some academics, financial risk has two components: the first is the risk that the company will not be able to pay its debts and obligations; the second is the danger that financial leverage factors would cause variations and fluctuations in share price earnings. One of the symptoms of financial risk is bankruptcy, which occurs automatically when a business becomes insolvent [8]. Many professionals and academics have debated and developed the study on financial forecasting and early warning models. Univariate financial models, multivariate financial models, multivariate logistic regression models, and artificial neural network forecasting models are the models that are frequently utilized in real-world applications. Among them, artificial neural networks have strong fault tolerance and low data requirements and can perfectly handle noisy and incomplete data by breaking through the limitations of traditional statistical methods [9]. Using the characteristics of self-learning, training, and simulation of neural networks, we can adapt to the changing business environment and analyze the financial management of enterprises to determine whether a predicted sample has financial risks.

Based on the above research background, the financial forecasting and early warning models of enterprises began to receive general attention. In order to address the system and methodological issues in the financial management of enterprises operating under the pandemic norm, this study makes an effort to employ a more rigorous and persuading approach. An enterprise financial forecasting model is built by examining and utilizing LSTM networks to address the financial forecasting issue. Enterprise financial history data are fed into the model repeatedly for training, after which the predicted enterprise financial trend is realized [10].

## 2. Related Works

### 2.1. The Impact of the Epidemic on the Financial Management System of Enterprises

Financial management plays a key role for an enterprise. The basic activities of an enterprise consist of four parts. These five parts are investment, financing, operation, income, and expenditure. This division causes the further division of financial management into four parts. The first is investment management that mainly emphasizes on the capital expenditure of the enterprise. It includes investment to allocate assets for the enterprise which enables the enterprise to obtain higher productivity. The higher productivity then ultimately results into higher efficiency of the enterprise [10]. Secondly, financing management in order to expand business improves the internal management and other needs of enterprises to raise reasonable funds. For better fund raising, it is therefore necessary for enterprises to carry out financing management. Third is working capital management, which mainly manages the working capital and current liabilities of the enterprise [11]. And lastly, through the implementation of income and expenditure management, income and expenditure management can reasonably control and adjust all the economic business transactions and transactions of the whole enterprise. It also reasonably allocates the revenue of the enterprise.

It is a difficult task to integrate the financial information and related data of an enterprise to better serve the management and decision making of an enterprise through scientific and effective implementation of reasonable enterprise capital management [12]. But a major premise needed is to take information technology as the basis, so that enterprise financial data and related information can be integrated with modern information system platform. As a result, enterprises can obtain relevant information and data more systematically and accurately.

The dilemma faced by enterprise finance in the context of the epidemic includes the following four directions:

- Business income of enterprises: the first thing that declined is the impact of shutdown and production suspension. Except a very small number of enterprises such as mask manufacturers, most of the remaining enterprises are stuck in the situation of shutdown and it is difficult to resume work and production
- Increase in production costs: whether it is due to a sudden public event or the impact caused by the new crown epidemic, the effect on the production and operation of the enterprise is huge [13]. The instability in the prices of raw material also makes the production cost of enterprises unstable. The production is, therefore, affected from two aspects
- Difficulty of enterprise capital turnover: different economic situations will have different impacts on the capital turnover of enterprises. Due to the new crown epidemic, the government departments and some related enterprises will put more energy on the prevention and control of the epidemic. Therefore, the debt clearing task of the enterprise cannot be effectively implemented and completed
- Increased pressure of industrial adjustment: in the new situation of the epidemic, enterprises want to seek development and find a way out. They also seek to adjust their industrial structure and change their development strategy. Enterprises must choose this as a road to adopt [14]

The outbreak of the new crown epidemic has affected the public safety of the society. It has restricted the development of the market economy. The development of the enterprise is also at serious setback. Under the impact of the new crown epidemic, companies need to better coordinate all financial relationships, sound financial budgets and strengthen capital management. It also needs controlled labor costs and raw materials and with open source and cut costs [15].

### 2.2. Current Status of Financial Forecasting Model Research

Through study and business managers' practical knowledge of financial control in day-to-day operations, academics have offered several qualitative methods for enterprise financial forecasting. These methods include the four-stage symptom analysis method [16], the flow chart method, the analytical survey method, and the management scoring method. Despite the relatively late start of the domestic research, a number of excellent research findings have emerged, and deeper investigation and analysis of connected themes have been carried out.

The models used for corporate financial forecasting have evolved from univariate forecasting methods to multivariate forecasting methods. The application of conditional probability models such as logistic models has further improved the performance and prediction accuracy of multivariate models [17]. Artificial neural network models have been used to corporate financial forecasting in recent years in the context of big data technology and machine learning sweeping in the world. This shows better performance and increased predicting accuracy. These models include univariate model, multivariate model, discriminant analysis model, multivariate linear model, and artificial neural network model. Models are given below with detailed description.

- Univariate models: based on this, some researchers continued to investigate the discriminative power of univariate model on financial crises and were the first to construct financial evaluation prediction models using statistical methods. It was concluded that the three best indicators for predicting the financial condition of a company are the total cash-to-debt ratio, the gearing ratio, and the net profit margin of total assets
- Multivariate model: the earliest multivariate models were the *Z* model and the ZETA model. ZETA model was developed from the *Z* model. The earliest study of corporate finance using multivariate linear discriminant models was the *Z* model, which applied multiple discriminant variables to corporate finance forecasting models. This model collected data on five financial indicators from 33 failed companies and 33 normal companies of the same size in the manufacturing industry. It constructed a *Z* model that can be used to predict whether a company is in financial crisis by using a comprehensive weighted average. Based on the *Z* model, a researcher conducted a more in-depth study and obtained a modified ZETA model [18]
- Discriminant analysis model: the discriminant analysis is a technique for statistical identification and analysis and is used in financial forecasting. It establishes the discriminant function by using samples with known actual classification and measured observations of each indicator as training samples. The previous *Z* model and ZETA model are in fact a simple multivariate linear discriminant model. But discriminant analysis is not limited to this, and there are many other methods of discriminant such as maximum likelihood, distance discriminant, canonical discriminant, and Bayes discriminant
- Multivariate linear model: subsequently, domestic scholars have also adopted logistic model as a method of enterprise financial evaluation. Some researchers have used logistic model to study the financial status of agricultural enterprises after factor analysis of variable indicators and constructed an industry financial evaluation model. Based on this, a researcher used logistic regression to construct a bank financial measurement model with comprehensive monitoring of multiple indicators [19]. Other researchers added financial indicators to the financial forecasting index system and used *Z*-value model and logistic regression model. By comparing the results of the two financial forecasting models, it was found that the method using logistic regression has a higher accuracy rate than the *Z*-value model
- Artificial neural network model: in recent years, the artificial neural network model has attracted more attention and has become a newcomer in the enterprise financial forecasting model [20]. Applying the classification method of neural network to the prediction and evaluation, the enterprise finance forms the artificial neural network model of prediction

### 2.3. Current Status of Research on Financial Risk Early Warning Model

Foreign security markets are established earlier, and scholars there are more mature in financial early warning research than in China. The study of financial risks from several aspects is shown in Figure 2. In China, the study on early warning systems for financial crises is still in the embryonic stage. Despite the large number of literature, the majority of it suffers from several issues. These issues include the use of nonparametric methods. It is also challenging to reflect the complete image of an enterprise's financial state due to the lack of comprehensiveness in financial data.

We must create an integrated framework of “digital technology and traditional management tools” in terms of management tools. Management tools are the means and technologies to conduct financial activities. The use of digital technology by financial activities of enterprises is used as a means to develop ports and analysis systems to connect with business and the outside environment, to establish a new material foundation for information integration and resource allocation of financial activities, and to realize strategies and goals of digital transformation and value sharing. These all are required in order to realize digital transformation and deep integration of business and finance [21]. On the one hand, the traditional management tools such as SWOT can be used to help you understand your business. On the other hand, some other traditional management tools such as comprehensive budgeting, DuPont analysis system, balanced scorecard, job costing, and other management ideas and economic principles are not obsolete and can still play a role in making financial and business decisions to improve the efficiency, analysis, and forecasting ability with the help of digital technology [22]. Therefore, it is necessary to integrate digital technologies with traditional management tools to form a unified framework for their use. As a result, the technical means of financial activities can meet business requirements and become more comprehensive and efficient.

BP neural network method is recognized and widely used by many scholars. The BP neural network algorithm is a nonlinear mapping model which can handle experimental data with high correlation between indicators or incomplete data and produce better prediction results [23]. Compared with traditional statistical methods, BP neural network has its incomparable advantages: (1) in terms of model prediction, the BP neural network model has higher accuracy in predicting financial distress. (2) In terms of sample selection, the BP neural network model does not require the overall sample to obey a particular distribution, thus reducing the difficulty in sample selection and expanding the scope of the research object. (3) The BP neural network model can be set to a smaller size [24]. The BP neural network model can set a small systematic error. The system can find the intrinsic connection between input and output through the learning and training process based on the sample data and make self-correction according to the requirement of systematic error.

In short, it overcomes the limitations of traditional statistical methods to a certain extent and has the ability of fault tolerance and powerful functions of processing information. It is also capable of training of data information so as to predict the future financial situation.

## 3. Algorithm Design

### 3.1. LSTM-Based Financial Forecasting Model

In this section, an LSTM forecasting model is established. The model is established by adding temporal attributes in financial data to the existing forecasting model through the spatiotemporal dependencies between the starting and ending positions in the obtained enterprise financial data. Since the volume of enterprise financial data is influenced by working day and nonworking day factors, it has a strong cyclical pattern. Therefore, by studying and analyzing the data in the previous time period, it is possible to forecast the financial trends in the subsequent period [25]. The construction steps of the financial forecasting model are divided into various points given below.

- Data preprocessing: prior to being smoothed and normalized, the historical financial data are first cleaned and their noise level is decreased. By determining whether the original data is volatile, this method is used to lower its volatility
- Using spatiotemporal clustering, the original data are categorized, and the data are then divided according to the categorization outcomes
- Choosing the proper activation function, defining the values of variables like learning rate, and the maximum number of iterations are some examples of ideal neural network parameters
- Training of the model: until the design criterion of the minimal gradient error calculation function is fully satisfied, the gradient weight function is updated using the minimum gradient error calculation function
- Validate the model effect: financial data are special in that they depend on whether it is a working day as well as the historical time at which they were collected

The framework of the financial forecasting model constructed in this paper is schematically shown in Figure 3. The model first divides the financial data into 12 times series according to one day; then, the original data is divided by a quadratic spatiotemporal clustering algorithm combining ST-DBSCAN and *K*-means. The time series and spatial attributes are input as information into the prediction model of LSTM neural network which can be obtained by analyzing and training a large amount of historical information [26]. As a result, the prediction model based on quadratic spatiotemporal clustering and LSTM neural network is obtained.

A unique type of RNN network called LSTM has distinct forgetting and memory patterns. In the present traditional machine learning analysis methods, it can accurately study and determine the temporal properties of a large amount of data. As a result, it effectively reduces the data gradient explosion and disappearance in the present standard neural network prediction models. Three fully connected layer modules with distinct roles construct the LSTM neural network. These layers are called forgetting gate, input gate, and output gate. The “gate structure,” which is intended to successfully achieve the objective of information control, allows each neuron to transfer information to each other in a selected manner [27]. The training of the models in LSTM neural networks is based on the backpropagation principle, just like in RNN neural networks.

The difference is that when the parameters of the backpropagation process are updated in the network, as shown in Figure 4, the backpropagation direction of the error in the LSTM network has two main directions. One is the backpropagation direction along the point in time in the network and the other direction is the backpropagation of the corresponding error term to the previous layer. According to the corresponding error term, it is to calculate the gradient between the weights [28]. The other direction is to backpropagate the corresponding error terms to the next level and calculate the gradient between the weights according to the corresponding error terms.

Since LSTM is characterized by using historical data to “trace back,” if the historical data is insufficient, the gradient will disappear. Choosing a better activation function and changing the propagation structure are the common solutions to “gradient disappearance.”

The activation function is often used in the training process, and sigmoid is often used as the activation function for deep neural networks. However, problems such as gradient disappearance can easily occur during this function. This problem can cause the weights of the layers to disappear during the training process and can no longer change. Only the data are weighted by the fixed weights causing interference to the training of the neural network [29, 30]. Deep neural networks have similar timing with LSTM. However, to avoid the occurrence of similar gradient disappearance in LSTM networks, this paper uses the ReLU activation function.

The loss function is the mean square error (MSE). It is a loss function representing the error between the actual output and the expected output of a neural network and is calculated as follows:

(1) $$\begin{array}{c} \text{MSE}=\frac{1}{n}\overset{n}{\underset{i=1}{\sum }}{\left(y-y^{\prime }\right)}^{2}, \end{array}$$

where the sample size is *n* and the expected value is *y*.

For the stochastic gradient descent algorithm, it is no longer necessary to have all the samples undergo gradient computation during the gradient descent of the network. Parameters are, however, updated based on the results of each execution of the training. The formula for gradient descent is shown as

(2) $$\begin{array}{c} x_{t+1}=x_{t}-\eta \nabla f\left(x_{i}\right) \end{array}$$

Neural networks learn faster by using stochastic gradient descent as the optimization function, i.e., faster convergence of the loss function.

### 3.2. Financial Risk Early Warning Model Based on BP Neural Network

The learning process of the model is shown in Figure 5. The learning samples are added in the input layer, and the data are processed in the implicit layer through forward transfer. The values are then passed to the output layer nodes under the joint action of weights, thresholds, and activation functions [31]. In the output layer, the actual value is compared with the expected value. If there is a large error and the expected accuracy is not reached, the model algorithm enters the reverse transfer stage and continuously adjusts to make the output value as close to the expected value as possible.

The number of nodes in the implicit layer of the model is complicated to determine and is generally set by empirical values which is based on the sample size and the number of variables [32]. Therefore, the number of nodes in the implicit layer is set as follows:

(3) $$\begin{array}{c} L=\sqrt{m+n}+a, \end{array}$$

where *m* is the number of input nodes, *n* is the number of output nodes, and *a* is any constant between 1 and 10.

Correction weights using the general error in the implied layer and the input vector in the input layer are as under:

(4) $$\begin{array}{c} w_{ij}\left(N+1\right)=w_{ij}\left(N\right)+\beta \cdot e_{j}\cdot x_{i},\\ \theta_{j}\left(N+1\right)=\theta_{j}\left(N\right)+\beta \cdot e_{j}. \end{array}$$

The neural network would not be able to produce the convergence effect if there are more learnings than the set number.

## 4. Experiment

### 4.1. Experimental Results of Financial Prediction

First, the neural network training results are analyzed. The financial prediction model based on the LSTM neural network has a gradually decreasing loss value because the amount of data increases as shown in Figure 6. Although the data volume is large and the data features are complex, the loss function is not high and can remain stable. The model is trained 10 times, and the loss value of the prediction model gradually stabilizes when the model is trained to a certain degree. The loss value does not decrease with the increase of the number of times the model is trained, so that the gradient of the model in the training process can be effectively avoided to disappear.

Then, the same input information, number of network layers, loss function, and optimization algorithm were used for the prediction models of BP, RNN, and LSTM, respectively. To reduce random errors, each model parameter was carefully tuned separately and tested five times. The final average results are shown in Figure 7. The prediction results obtained using the LSTM neural network match the actual fold (green fold) more closely in the image when compared to the prediction results of the BP (red fold) and RNN (blue fold) network prediction models. This indicates better prediction results.

### 4.2. Experimental Results of Financial Risk Early Warning

The training fit sample is the first 100 data for model training, and the prediction test sample is the last 40 data. The model is validated with the data. If the result is good, the established early warning model is proved to be excellent.

The number of nodes in the implied layer was solved several times according to the above formula. The model was tested in order to find the best fit when the implied layer was 8 according to the error size. The sample training and actual comparison is shown in Figure 8. The fitting result of BP neural network can be considered to be optimal at this time. The fitting result for the enterprise financial warning results reached 97%. The difference between the actual value of 40 data and the target desired output is not significant.

Based on the above verification of the continuous adjustment of the nodes in the implicit layer, it can be concluded that the best accuracy of model fitting was achieved when the number of implicit nodes was set to 8 for the early warning model using the BP neural network. The prediction results for each early warning interval are shown in Table 1. Table 1 shows that the accuracy of model fitting reaches 97.66% and the prediction accuracy is 96.35%. The model results at this time have the highest accuracy and the least training times.

In this paper, three models are applied in practice as financial early warning models for enterprises and the experimental results are shown in Table 2. According to the results of the prediction test, it was found that the prediction effect of the logistic model of financial indexes and the logistic model of comprehensive indexes were in the better interval, 92.34% and 91.08%, respectively. However, the prediction effect of BP neural network was excellent. The integrated logistic model outperformed the logistic model with only financial indicators in terms of fitting and prediction results; however, both the logistic model with only financial indicators and the integrated logistic model with qualitative indicators were not as accurate as the BP neural network.

## 5. Conclusion

The new coronavirus epidemic is a sudden public health event that has caused the world economy to be hit hard. In this situation, the development of enterprises is also facing a huge survival test. In this context, it is important to discuss the financial management of enterprises under the epidemic as their resilience in the face of emergency can effectively reflect their financial management level. In this paper, we propose a system that can automatically predict financial trends and provide early warning of financial risks by combining artificial neural networks with the current difficulties faced by enterprises in the new situation. According to the wide application of machine learning in the field of data mining, this paper constructs a financial prediction model by using the LSTM neural network. By training and learning the enterprise financial data set with different spatial and temporal attributes of data attributes, the future financial trend of the enterprise is finally derived. Then, a BP neural network is combined with the enterprise risk warning model, and the results are obtained by training and learning the training samples for several times. The experimental results show that the LSTM-based prediction model can effectively predict the enterprise financial trends and has better results than BP and RNN neural networks. The results of risk prediction model based on BP neural network show a satisfactory impact in analysis of enterprise financial early warning. The attempt of study to apply artificial intelligence technology to enterprise financial management can provide some reference for enterprise financial management.

## Figures and Tables

**Figure 1:** Impact of the epidemic on economic activities.

**Figure 2:** Influencing factors of financial risk.

**Figure 3:** Flow chart of prediction model based on LSTM.

**Figure 4:** LSTM network structure diagram.

**Figure 5:** Structure of the BP neural network model.

**Figure 6:** LSTM prediction model based on the 10 times training loss curve.

**Figure 7:** Comparison of prediction of three kinds of neural networks.

**Figure 8:** Comparison between prediction and actual graph.

**Table 1:** Classification of predictive test results.

Observation value	Predictive value			Percentage correction
	Security	Mild	Severe	
Safety warning interval	31	2	1	95.83%
Mild warning interval	2	23	4	97.66%
Severe warning interval	0	0	7	93.47%
Total percentage	85.21%	76.43%	12.95%	96.35%

**Table 2:** Comparison of financial early warning model results.

Warning interval	Logistic model		BP model	
	Fitting	Predicting	Fitting	Predicting
Safety warning interval	92.34%	91.08%	96.27%	92.42%
Mild warning interval	86.75%	83.82%	91.63%	89.87%
Severe warning interval	90.31%	88.97%	92.49%	90.53%
Total percentage	89.62%	87.53%	90.82%	89.04%

## Data Availability

The datasets used during the current study are available from the corresponding author on reasonable request.
